# Application of deep neural network and deep reinforcement learning in wireless communication

This article has been retracted.

**DOI:** 10.1371/journal.pone.0235447

**Published:** 2020-07-02

**Authors:** Ming Li, Hui Li

**Affiliations:** National Intellectual Property Administration, Beijing City, China; University College London, UNITED KINGDOM

## Abstract

**Objective:**

To explore the application of deep neural networks (DNNs) and deep reinforcement learning (DRL) in wireless communication and accelerate the development of the wireless communication industry.

**Method:**

This study proposes a simple cognitive radio scenario consisting of only one primary user and one secondary user. The secondary user attempts to share spectrum resources with the primary user. An intelligent power algorithm model based on DNNs and DRL is constructed. Then, the MATLAB platform is utilized to simulate the model.

**Results:**

In the performance analysis of the algorithm model under different strategies, it is found that the second power control strategy is more conservative than the first. In the loss function, the second power control strategy has experienced more iterations than the first. In terms of success rate, the second power control strategy has more iterations than the first. In the average number of transmissions, they show the same changing trend, but the success rate can reach 1. In comparison with the traditional distributed clustering and power control (DCPC) algorithm, it is obvious that the convergence rate of the algorithm in this research is higher. The proposed DQN algorithm based on DRL only needs several steps to achieve convergence, which verifies its effectiveness.

**Conclusion:**

By applying DNNs and DRL to model algorithms constructed in wireless scenarios, the success rate is higher and the convergence rate is faster, which can provide experimental basis for the improvement of later wireless communication networks.

## 1. Introduction

With the rapid development of science and technology, the development of mobile networks is faster than ever. For example, 5G networks have been commonly used in many first-tier cities, making people’s communication more convenient, which means that wireless communication technologies are widely used in reality. However, since a large number of wireless terminal devices are connected to the communication network, the wireless spectrum resources are becoming scarce [1,2]. Although wireless cellular technology has eased the spectrum problem in mobile communications, it is still insufficient to meet user capacity and cannot fundamentally solve the problem of people’s communication needs and spectrum shortage [3]. Therefore, how to rationally plan and apply the spectrum resources in wireless communication has become the focus of scientific researchers.

In the wireless communication network, the electromagnetic spectrum resources of the radio are very precious, and the government has also rationally allocated them. However, as the number of Internet of Things (IoT) terminals increases, the congestion situation still cannot be alleviated. But it doesn’t mean that the resources have been exhausted. Studies have shown that up to 70% of spectrum resources in some parts of the United States are idle most of the time, and the utilization rate of some of them is only 15% [4]. Through this research, it is verified that the current spectrum resources of various countries have not been used reasonably [5]. thus, the National Spectrum Supervision Bureau has managed this issue. According to the original traditional electrostatic allocation mechanism, only authorized users can communicate in the specified frequency band. Also, for dynamic spectrum resource allocation, unlicensed users and authorized users are allowed to share the current frequency band. However, as the utilization of spectrum resources by authorized users changes over time, non-authorized users need to intelligently sense the current frequency band usage [6]. Therefore, choosing a reasonable time and communicating with appropriate power to maximize the utilization of spectrum resources and finally alleviating the pressure of insufficient spectrum resources have become the problems that need to be urgently solved at present. Reinforcement learning, as a new emerging technology, has great advantages in environmental automatic exploration and self-decision, and also has great potential in solving dynamic resource allocation problems [7]. With the popularity of deep learning algorithms in the computer field, the concept of deep reinforcement learning (DRL) has been proposed. Compared with traditional reinforcement learning algorithms that can only observe low-dimensional features, DRL can train the obtained agents to learn the actions in images or videos by observing high-dimensional raw data [8,9]. Generally, DRL has two characteristics. The first is that its optimization goal is the long-term return of the system rather than the immediate return. The second is that the application process does not require prior information about the environment to achieve approximate optimal performance, which has autonomous exploration and optimal decision-making capabilities [10]. Therefore, it is of great practical significance to introduce DRL into wireless communication technology.

In summary, as an emerging technology, there is not much research on DRL in the field of wireless communication. Therefore, in the future, to alleviate the pressure of spectrum usage in wireless communication, based on the characteristics of DRL, this study applies DRL to wireless communication networks. An intelligent power algorithm model based on deep neural networks (DNNs) and DRL is constructed, and the model is simulated in MATLAB to verify its effectiveness, which provides experimental ideas for the later development of the wireless communication field.

## 2. Literature review

With the increasing popularity of mobile network applications, the development of wireless communication technology has been accelerated. Many scholars have conducted research on its performance and improvements. Huang et al. [11] proposed a hybrid optical wireless network based on free-space optic (FSO)/visible light communication (VLC) heterogeneous interconnection for the future air-ground-sea integrated communication architecture, especially in an environment that was radio frequency-sensitive or under safety requirements. In addition, three basic network mechanisms were designed to evaluate their performance. Finally, it was found that VLC at different speeds and FSO under five typical air quality conditions had good transmission performance, and the feasibility of this hybrid optical wireless network was verified [11]. To improve the radiation quality of the receiving line, Nayak et al. [12] simplified the control of wave speed, shape, and directionality, and helped the overall implementation of the framework. By introducing the current status of improvements in telecommunication frameworks and radio lines, some schemes of the receiving equipment were envisaged. Then, the forward direction and important components compatible with the existing communication framework were decomposed, and the structural adjustment and mode of the receiving device were analyzed. Finally, it was found that the antenna mainly used a flat structure, which provided great convenience for the integration and miniaturization of mobile terminals [12]. Sopara et al. [13] conducted a comparative study of energy-saving communication schemes for wireless sensor networks (WSNs); finally, it was found that the proposed scheme had good energy-saving effects and provided an experimental basis for the improvement of wireless communication technology [13].

In the era of the IoT, people face massive amounts of data and information every day. Therefore, the intelligent processing of data plays a vital role. Deep learning is used for intelligent extraction of information features, and its applications in all walks of life are becoming increasingly widespread. In the field of materials medicine, Ohsugi et al. [14] applied deep learning to the detection of rhegmatogenous retinal detachment (RRD) in ultra-wide field fundus images; eventually. they found that the diagnostic accuracy of RRD with ultra-wide field fundus increased significantly, which was critical for the early diagnosis of RRD and prevention of blindness [14]. In the field of logistics, Sremac et al. [15] applied deep learning to the construction of AI-adaptive neural fuzzy logistics system models; eventually, they found that the model had better accuracy in the logistics chain and could be flexibly applied to supply chain management of various types of products [15]. In the medical field, Wu et al. [16] applied deep learning to the three-dimensional reconstruction of digital holographic microscope models; by comparing with traditional bright-field microscopic images, they found that the wave propagation frame of hologram could achieve fast three-dimensional imaging of bright-field contrast objects in a single hologram [16]. In the field of wireless sensing, Leong et al. [17] studied the scheduling of sensor transmissions to estimate the status of multiple remote dynamic processes, and proposed a relevant Markov decision process (MDP); then, by using deep Q-network (a new DRL algorithm) to solve the MDP, it was found that the proposed algorithm significantly outperformed the existing algorithms [17]. In terms of deep neural networks (DNNs), Chen et al. [18] explored the anti-noise ability of DNNs. By proposing a new activation function rand-softplus (RSP) to simulate the response process, the anti-noise ability of DNNs has been improved accordingly [18]. Joy et al. [19] used DNNs as regression models. Through the training and optimization of the model, it was found that the method based on DNNs can achieve the standardization at the discourse level [19]. Liu and Wang [20] used DNNs to model the probabilistic pitch state of two simultaneous speakers. Also, they proposed two different training strategies of DNNs, expanding the application of DNNs in the field of language and signal processing [20]. Dai et al. [21] introduced a synthesis tool NeST to supplement network pruning during the training process to learn weights and compact DNN structures, thereby achieving optimization of the DNNs architecture [21].

In summary, there are many researches on DRL and wireless communication; however, studies combining DRL and DNNs with wireless communication technology are rare. Therefore, to improve the performance of wireless communication technology, this study applies DNNs and DRL algorithms to wireless networks, providing experimental basis for the development of the wireless communication industry.

## 3. Methods

### 3.1. Wireless communication network

Wireless communication network technology is a technology that uses electromagnetic waves as a medium to communicate in free space. Its principle is to modulate the information to be transmitted to the radio wave band through a carrier with a higher frequency and send it out through the antenna of the transmitter, thereby realizing the transmission of information. Usually, electromagnetic waves travel through free space to reach the receiving end’s antenna, and the receiving end recovers the original information through demodulation. The architecture of wireless communication networks often requires many different types of key technical support, including software-defined network (SDN) technology, information center network (ICN) technology, D2D (Device—to—Device Communication) communication technology, and wireless network virtualization (WNV) technology [22,23]. A typical communication-cache system for a wireless communication network is shown in Fig 1.

**Fig 1:** Schematic diagram of a typical communication-cache system for a wireless communication network.

Heterogeneous networks are one of the main architectures for the development of wireless communication networks. Usually, small cellular base stations are deployed in a small area to enhance the coverage of macro cellular base stations. However, the utilization of small cellular base station buffers still requires radio access network (RAN) to transmit traffic [24,25]. Although D2D communication technology allows users to share contents, compared with small cellular base stations, the storage capacity of user equipment is small, the battery capacity is limited, and the cost is high. Therefore, the framework mainly covers D2D, multi-hop D2D, cooperative D2D, direct small cellular base stations, and small cellular base stations, which are typical paradigms. The D2D cache-communication paradigm mainly means that a user equipment obtains content from other user equipment in its vicinity through D2D communication, thereby improving the user service quality between different cells. The multi-hop D2D cache-communication paradigm mainly uses adjacent user equipment as a relay to access the small cellular base stations in other cells to retrieve content, allowing for more extensive collaborative caching and delivery and improving resource utilization. The collaborative D2D cache-communication paradigm refers to a D2D transmission method for collaboration when a copy of a content is cached on multiple user devices. Direct small cellular base station cache-communication paradigm means that when the required content is not pre-cached in the adjacent user equipment, the requester can also request the content directly from the connected small cellular base station, which finally achieves lower latency. The cooperative small cellular base station cache-communication paradigm means that when content required by a user equipment is not cached to an adjacent small cellular base station, a virtual connection is established with the user device to obtain the required content from other small cellular base stations.

### 3.2. DNNs

DNNs, as a new research area, have developed rapidly. Currently, DNNs have formed different models, mainly including generative models, discriminative models, and hybrid models. In the DNNs structure, different connection rules correspond to different network structures, such as fully connected network, which is a multilayer feed-forward neural network. It consists of an input layer, a hidden layer, and an output layer. In addition, each neuron in the latter layer is connected by all neurons in the previous layer. The classic structure is shown in Fig 2 [26].

**Fig 2:** Structure of DNNs.

As shown in Fig 2, each circle represents a neuron. The neurons in the output layer function as a receiving container. The neurons in the hidden layer and the output layer represent neurons with activation function functions. The arrows indicate flow directions of information. The hidden layer in the figure includes two layers, and the number of hidden layers can be any non-negative integer in practice. In this study, the restricted Boltzmann machine (RBM) DNNs in generative models is mainly analyzed.

The RBM model is a special type of Markov random field. Its upper layer is a random hidden unit and can be regarded as some feature extractors. The lower layer is a random visible or observable unit layer. RBM can also be viewed as a bipartite graph, with one layer as the visual input layer (*v*) and one layer as the hidden layer (*h*); usually, the nodes between the same layers are not connected to each other [27]. The vectors *v* and *h* are set as the states of the input layer and the hidden layer, respectively. The state of the *i*-th node of *v* is represented by *v*_*i*_, and the state of the *j*-th node of *h* is represented by *h*_*j*_. The energy equation of the RBM model is as follows:

$$E(v,h|\theta )=-\sum_{i=1}^{n}a_{i}v_{i}-\sum_{j=1}^{m}b_{j}h_{j}-\sum_{i=1}^{n}\sum_{j=1}^{m}v_{i}w_{ij}h_{j}$$ (1)

Where: *θ* = {*w*_*ij*_,*a*_*i*_,*b*_*j*_} is the RMB parameter, *w*_*ij*_ refers to the weight between the *i*-th node of the visible input layer and the *j*-th node of the hidden layer, and *a*_*i*_ and *b*_*j*_ quantities *v* and *h* refer to the *i*-th node of the visible input layer and the *j*-th node of the hidden layer. Therefore, when the three nodes are determined, the following probability equation can be derived:

$$P(v,h|\theta )=\frac{e^{-E(v,h|\theta )}}{Z(\theta )}$$ (2)

$$Z(\theta )=\sum_{v,h}e^{-E(v,h|\theta )}$$ (3)

In Eq (2), *Z*(*θ*) is the normalization factor. According to Eq (3), the distribution *P*(*v*|*θ*) of the observation data *v* is the focus of attention, which is often referred to as the likelihood function:

$$P(v|\theta )=\frac{1}{Z(\theta )}\sum_{h}e^{-E(v,h|\theta )}$$ (4)

When the state of the visible layer is determined, the nodes of the hidden layer are independent of each other, and it can be inferred that:

$$P(v|\theta )=\prod_{j}P(h_{j}|v)$$ (5)

The activation probability of the hidden layer at this time is:

$$P(h_{j}=1|v)=\sigma \left(b_{j}+\sum_{i=1}^{n}v_{i}w_{ij}\right)$$ (6)

$$\sigma (x)=\frac{1}{1+e^{-x}}$$ (7)

Where: *σ*(*x*) is the activation function. Since the visible input layer and hidden layer of RBM are symmetrical, when the state of the hidden layer is determined, the nodes of the visible input layer are independent of each other, and the following equation can be obtained:

$$P(v|h)=\prod_{i}P(v_{i}|h)$$ (8)

$$P(v_{i}=1|h)=\sigma \left(a_{i}+\sum_{j=1}^{m}w_{ij}h_{j}\right)$$ (9)

Given a sample set *D* = {*v*^(1)^,*v*^(2)^,⋯,*v*^(N)^} that satisfies the independent and identical distribution, the parameter *θ* = {*w*_*ij*_,*a*_*i*_,*b*_*j*_} needs to be learned. Then, the log-likelihood function is:

$$L(\theta )=\frac{1}{N}\sum_{n=1}^{N}\log P_{\theta }(v^{\left(n\right)})-\frac{\lambda }{N}{\left\|W\right\|}_{F}^{2}$$ (10)

The derivative of the log-likelihood function can be calculated to calculate the value of the parameter W when the log-likelihood function takes its maximum value.

$$\frac{\partial L(\theta )}{\partial W_{ij}}=E_{P_{data}}\left[v_{i}h_{j}\right]-E_{P_{\theta }}\left[v_{i}h_{j}\right]-\frac{2\lambda }{N}W_{ij}$$ (11)

Compared with a direct model with a hidden layer function, the RBM model has two advantages. One is that the model is simple in reasoning, and the hidden distribution of each hidden layer is multiplied to obtain the posterior distribution of the hidden layer. The second is to use multiple RBM is connected, and each layer of the deep network is easier to learn and obtain.

### 3.3. DRL

DRL consists of two modules: deep learning and reinforcement learning. It uses deep learning to extract features from complex high-dimensional data, transforms them into a low-dimensional feature space, and inputs them into reinforcement learning for decision-making. Typical DRL algorithms include deep Q-learning algorithms, deep strategy gradient algorithms, and asynchronous dominant Actor-Critic algorithms. In this study, the classic deep Q-learning algorithm is mainly used. Usually, a reinforcement learning problem includes elements such as state, action, reward, state transition probability, strategy, and value function [28]. Reinforcement learning problems can usually be described as the optimal control of the MDP. However, it is not necessary to know the state space, transition probability, and reward function. An MDP can consist of a limited number of states, actions, and rewards, and can be expressed as:

$$x_{0},a_{0},r_{1},x_{1},a_{1},r_{2},x_{2},a_{2},r_{3},\cdots ,x_{n-1},a_{n-1},r_{n},x_{n}$$ (12)

Where: *x*_*j*_ indicates the state, *a*_*j*_ indicates action, *r*_*j+1*_ indicates the reward after taking actions. When the state reaches a preset termination state *x*_*n*_, one MDP ends. Reinforcement learning usually includes trial and error search and delayed reward. Q-learning algorithm, as one of the most widely used model-free reinforcement learning algorithms, can be implemented by a lookup table or a function approximator, or sometimes a non-linear approximator, such as a neural network or more complex DNNs. The Q learning algorithm combined with DNNs is the deep Q learning algorithm [29]. *X* = {*x*_1_,*x*_2_,⋯,*x*_*n*_} is set as the state space and *A* = {*a*_1_,*a*_2_,⋯,*a*_*m*_} is the action space. Based on the current state *x*(*t*)∈*X*, the agent selects an action *a*(*t*)∈*A* to act on the environment. The reward when the environment changes to a new state *P*_*x*(*t*)*x*(*t*+1)_(*a*) according to a certain state transition probability *x*(*t*+1)∈*X* is recorded as *r*(*x*(*t*),*a*(*t*)). The cumulative discount reward available at state *x* is a function of the state value expressed as:

$$V^{\pi }(x)=E\left[\sum_{t=0}^{\infty }\varepsilon^{t}r(x(t),a(t)|x(0)=x)\right]$$ (13)

Where: E is the mathematical expectation, and *ε* is a discount factor with a range of *ε*, which considers an infinite time range. According to the nature of the Markov chain, the state at the next time point is determined only by the current state, and has nothing to do with the previous state.

$$V^{\pi }(x)=R\left(x,\pi (x)\right)+\varepsilon \sum_{x'\in X}P_{xx'}(\pi (x))V^{\pi }(x')$$ (14)

Where: *R*(*x*,*π*(*x*)) is the average of instant reward *r*(*x*,*π*(*x*)), and *P*_*xx*'_(*π*(*x*)) is the state transition probability from state *x* to *x’* after performing action *π*(*x*). When the reward R and transition probability P are unknown, the Q learning algorithm is the most widely used method of obtaining strategy π*. The Q function can be defined as:

$$Q^{\pi }(x,a)=R\left(x,a\right)+\varepsilon \sum_{x'\in X}P_{xx'}(a)V^{\pi }(x')$$ (15)

Where: *Q*^*π*^(*x*,*a*) efers to the discount accumulation reward that can be obtained by continuing to execute the optimal strategy after performing the action a in the state *x*. Then, the largest Q function is:

$$Q^{\pi *}(x,a)=R\left(x,a\right)+\varepsilon \sum_{x'\in X}P_{xx'}(a)V^{\pi *}(x')$$ (16)

The cumulative status function of discounts can be written as:

$$V^{\pi *}(x)=\max_{a\in A}\left[Q^{\pi *}(x,a)\right]$$ (17)

It can be seen from the above equation that the goal of reinforcement learning can be changed from the optimal strategy to obtain the most suitable Q function. In practice, the Q function is often estimated by a function approximator, sometimes a non-linear approximation, such as neural network *Q*(*x*,*a*;*θ*)≈Q*(*x*,*a*), which is the Q network. Parameter *θ* refers to the weight of the neural network. The network is trained by adjusting *θ* in each iteration to reduce the mean square error [30].

### 3.4. Construction of intelligent power algorithm model

In this study, a simple cognitive radio network consisting of only one primary user and one secondary user is considered. In this wireless communication network, the primary user enjoys the priority use right of the current frequency band, that is, it can use spectrum resources according to its plan. The model is constructed in the hope that the secondary user will share spectrum resources with the primary user without causing harmful interference to the primary user and improve the utilization of the spectrum resources. This study assumes that the primary and secondary users update their respective transmit powers simultaneously in the same time frame, that is, the adjustment of the transmission power is considered based on a single time frame, and the time frame structures of the primary and secondary users are completely synchronized. For primary and secondary users, the measurement of service quality at the receiving end is mainly determined by their respective signal-to-noise ratios, and the signal strength in the environment is sampled and measured by sensors. To meet the quality of service requirements, the primary user sends its power based on an adaptive change of its power control strategy, while the secondary user’s appropriate power control algorithm mainly uses the deep Q network (DQN) in the DRL algorithm to replace Q-learning and learns the power control algorithm of the secondary user.

DNNs Q training requires a large amount of data, and reinforcement learning is different from traditional supervised machine learning. There is no ready-made training data; thus, the training data for the network in this study needs to be generated. The training of Q network can be realized by adjusting parameter *θ*. The training goal is to minimize the following loss function:

$$H(\theta )≜\frac{1}{\left|\Omega_{k}\right|}\sum_{i=\Omega_{k}}{\left(Q'(i)-Q(s(i),a(i);\theta )\right)}^{2}$$ (18)

Where: within *Q*(*s*(*i*),*a*(*i*);*θ*), *s*(*i*) is the state, *a*(*i*) is the action, Ω_*k*_ is the index set of the small batch of data randomly selected during the k-th iteration training, |Ω_*k*_| is the size of the data index set, and *Q*'(*i*) is the action obtained with the current parameters-value function, which is specifically expressed as:

$$Q'(i)=r(i)+\gamma \underset{d}{\max}Q(s(i+1),a';\theta_{0})$$ (19)

Where: *θ*_0_ represents the network parameters under the current iterative situation. This network parameter is different from other traditional supervised learning in that the target value Q in DQN learning will change with the change of network weight. The specific steps of the network algorithm are shown in Table 1.

**Table 1:** Flow of DQN algorithm for power control.

Algorithm name: DQN algorithm for power control
Initialize DNNs Q and set the weight as *θ*_0_.
Randomly initialize p_1_(1) and p_2_(1), and obtain s (1).
For k = 1 to K do
Obtain p_1_(k+1) according to the primary user’s power control update strategy.
The secondary user randomly selects an action with a probability of ε_k_ and a(k) with a probability of 1-ε_k_.
Obtain the state s(k+1) according to the random observation model, and observe the reward r(k).
Store data set *d*(*k*)≜{*s*(*k*),*a*(*k*),*r*(*k*),*s*(*k*+1)} in memory container D.
If k≥0 then
Randomly sample small sample set {*d*(*i*)|*i*∈Ω_*k*_} from memory container D, where Ω_*k*_ refers to the index set of small batch data randomly selected during the k-th iteration training.
Update *θ*_0_ by minimizing the loss function (Eq (18)).
End if
If s(k) is the ultimate state
Randomly initialize p_1_(k) and p_2_(k), and obtain s(k).
End if
End for

For the model algorithm proposed in this study, the MATLAB platform is used for simulation experiments, and TensorFlow is used as a deep learning library. In this system modeling, the parameter design includes the transmit power (unit: W) *P*_1_ = {0.05,0.1,⋯,0.4} and *P*_2_ = {0.05,0.1,⋯,0.4} of the primary and secondary users. The channel gain from the sender to the receiver of the primary and secondary users is 1, the noise power of the receiver is N_1_ = N_2_ = 0.01W, and the total number of iterations is set to K = 10^5^.

In the performance analysis, two power strategies are used for the primary user, and the specific parameters are set to Case 1 and Case 2 to analyze its loss function, success rate, and average number of transfers.

In Case 1, the primary user uses the first strategy method, with the number of sensors N = 10; the standard deviation of the random variable Wn(k) is used to calculate the shadow effect, and the measurement error is set to $\sigma_{n}=\left(p_{1}^{p}g_{1n}+p_{1}^{s}g_{2n}\right)/10$.

In Case 2, the primary user uses the second strategy method, with the number of sensors N = 10; the standard deviation of the random variable Wn(k) is used to calculate the shadow effect, and the measurement error is set to $\sigma_{n}=\left(p_{1}^{p}g_{1n}+p_{1}^{s}g_{2n}\right)/10$.

In addition, the DQN algorithm proposed in this study is compared with the traditional distributed clustering power control algorithm (DCPC) to analyze the performance of this study.

## 4. Results and discussion

### 4.1. Performance analysis of algorithm models under different strategies

By comparing the primary user’s loss function, success rate, and average number of transfers with the number of iterations k in the first and second power control strategies. The results are shown in Figs 3, 4 and 5. As shown in the figures, the two control strategies can learn effective power control strategies at the number of iterations of 10^3^ users. For the loss function, the second type of power control strategy has experienced more iterations than the first type. For the success rate, the second type of power control strategy has undergone more iterations than the first type of power control strategy. After a number of times, it can reach a state with a success rate of 1. For the average number of transfers, it is obvious that the second power control strategy requires more iterations to reach a stable state. Therefore, in the algorithm proposed in this study, the second power control strategy is more conservative than the first. In addition, the success rate of the algorithm model in this study can reach 1 under different strategies, which verifies its effectiveness.

**Fig 3:** Comparative analysis of the change of the loss function with the number of iterations k under different strategies.

**Fig 4:** Comparative analysis of the change in success rate with the number of iterations k under different strategies.

**Fig 5:** Comparative analysis of the results of the average number of transfers with the number of iterations k under different strategies.

Combined with the above analysis, it is obvious that the first power control strategy shows better performance in terms of loss function change, success rate change, or average transmission times and iteration times. In terms of the success rate index, both power control strategies are close to 100%, which indicates that the proposed algorithm model is effective and applicable. The combination of deep neural network and deep reinforcement learning shows great application potential in the field of wireless communication.

### 4.2. Performance comparison and analysis with other algorithms

To illustrate the advantages of the DQN algorithm proposed in this study, a comparative analysis is performed with the DCPC algorithm. As shown in the Fig 6, the primary and secondary users of the two schemes finally reach the convergence state. Meanwhile, the DQN proposed in this study can reach the final state after only a few conversion steps, and the optimization scheme of the DCPC algorithm has oscillations, which makes it take dozens of steps to reach convergence. Therefore, compared with the convergence of DCPC algorithm, it is obvious that the DQN algorithm based on DRL proposed in this study has obvious effectiveness.

**Fig 6:** Analysis of the change of the signal-to-noise ratio of the primary and secondary users with the state transition process.

The DRL algorithm includes the relevant content of deep neural network and deep reinforcement learning. It also means that the DQN algorithm based on DRL combines excellent performance in these two fields. The comparison with the DCPC algorithm also reflects it. The DQN algorithm based on DRL has stronger convergence. Thus, it is also more effective in the application of wireless communication.

## 5. Conclusions

This study addresses the practical problem of low frequency utilization in wireless communications and proposes a simple cognitive radio scenario consisting of only one primary user and one secondary user. The secondary user attempts to share spectrum resources with the primary user. An intelligent power algorithm model based on DRL is constructed. Then, the MATLAB platform is utilized to simulate the model. Finally, it is found that the success rate of the algorithm model can reach 1 when the main user adopts different strategies. The comparison with the DCPC algorithm shows that the convergence rate of the algorithm proposed in this study is higher, which verifies its effectiveness. Therefore, the proposed algorithm provides experimental basis for the improvement of wireless communication networks in the future. However, there are some shortcomings in the research process of this study. The algorithm proposed in this study only considers the situation of one primary user and one secondary user, but it is also common for multiple secondary users to coexist in real applications. Therefore, the power control of multiple secondary users will be the research direction of the subsequent study.

## Supporting information

S1 Data (XLS)

S2 Data (RAR)
